The article "Construction of Teaching Mode of Film and TV Art in Institution of Higher Learning Using Virtual Simulation Technology" was retracted in 2023. Reasons: suspected computer-generated content; unreliable results or conclusions; concerns about the data; concerns about the results or conclusions.

# Construction of Teaching Mode of Film and TV Art in Institution of Higher Learning Using Virtual Simulation Technology

**DOI:** 10.1155/2022/6216232

**Published:** 2022-07-04

**Authors:** Wei Xiong

**Affiliations:** College of Communication Science and Art, Chengdu University of Technology, Chengdu 610059, China

## Abstract

The modernization of education necessitates the enhancement of instructional quality. This paper begins with a basic overview of the current state of film and television art education and then goes on to examine the current state of film and television art education and develop a virtual simulation-based teaching mode for film and television art. This paper develops an instructional quality evaluation model to assess the feasibility of this teaching mode. In this model, GA is used to optimize BPNN's initial weights and thresholds, reducing the time it takes BPNN to find the weights and thresholds that satisfy the training termination conditions. Improve BPNN's prediction accuracy and convergence speed in relation to instructional quality evaluation results. The evaluation accuracy of this algorithm can reach 94.31 percent, which is 6.35 percent higher than other methods. Furthermore, the use of virtual simulation technology in the teaching of film and television art in higher education institutions can have a significant impact and have far-reaching research implications. The findings of this study can be used to improve the teaching of film and television art in institutions of higher learning.

## 1. Introduction

There are many new changes in the development of film and television art education at the moment, and the traditional teaching mode of higher art colleges cannot fully adapt to these changes. As a result, we must accelerate the construction of the teaching mode of film and television art [1]. Virtual technology is a brand-new science and technology concept. It creates a virtual space by combining computer simulation, computer graphics, man-machine interface, Internet, multimedia, and other technologies to provide the experiencer with a multidimensional sensory experience that includes sight, hearing, and touch [2]. Virtual experiment teaching is a new online teaching method that focuses on fidelity and immersion. Virtual experiment teaching can help solve some of the problems that traditional teaching has, as well as promote students' autonomy and inquiry learning. Using virtual simulation technology in art design classes can help students absorb knowledge and content more effectively [3]. Virtual technology stimulates students' learning enthusiasm and improves learning quality by providing new teaching ideas for virtual teaching. For students majoring in film and television media arts, virtual simulation experiment teaching can improve not only their intuitive feeling of the operating objects, but also their perception of teaching knowledge [4]. Film and television art as a major at a university is a relatively new discipline. This paper begins with an overview of the current state of film and television art education in China and then examines the measures taken to build the film and television art teaching mode, with the goal of making recommendations for the future development of film and television art education.

The article "Construction of Teaching Mode of Film and TV Art in Institution of Higher Learning Using Virtual Simulation Technology" was retracted in 2023. Reasons: suspected computer-generated content; unreliable results or conclusions; concerns about the data; concerns about the results or conclusions.

The evaluation of instructional quality is an important part of teaching management in institutions of higher learning, and the management of instructional quality is the key content of students' total quality management system. Instructional quality evaluation's scientificity, rationality, and timeliness are all important factors in improving instructional quality. However, because of its fuzziness, it is difficult to quantify, which adds to the complexity and difficulty of evaluating instructional quality. The gray system, analytic hierarchy process, fuzzy comprehensive evaluation, and cluster analysis [5, 6] are currently the most common methods of evaluating instructional quality in institutions of higher learning. These methods can essentially account for all types of factors that affect instructional quality, but they still have some flaws. Back propagation neural network (BPNN) [7] is an iterative algorithm that involves two processes: forward propagation of the input vector and backward propagation of the error. However, BPNN has the following drawbacks: it is easy to run into problems with local optimization, hidden layer determination, and recognition accuracy. The genetic algorithm (GA) is a computer program that models and simulates biological genetic mechanisms and natural selection. The problem solution can be evolved in the competition through “survival of the fittest,” resulting in a satisfactory solution to the problem. As a result, this paper employs GA to improve BPNN in order to construct an instructional quality evaluation model, which provides a feasible scheme for assessing instructional quality in higher education institutions. This paper mainly makes a relatively in-depth research on the construction of teaching mode of film and TV art in institution of higher learning based on virtual simulation technology, and its innovation lies in the following:

① Through the analysis of relevant data, this paper can know the theoretical concept of virtual simulation technology and its significance for students' teaching. At the same time, according to the existing problems, the corresponding solutions are put forward, and the teaching mode of film and TV art in institution of higher learning based on virtual simulation technology is constructed. Aiming at this teaching mode, this paper constructs an instructional quality evaluation model to evaluate the feasibility of this teaching mode.
② Aiming at the nonlinear characteristics of instructional quality evaluation and many nonquantitative factors in the instructional quality evaluation system, this paper establishes an instructional quality evaluation model. Aiming at the shortcomings of traditional BPNN, GA is used to optimize the initial weights and thresholds of BPNN, which reduces the time for BPNN to find the weights and thresholds that meet the training termination conditions. Further improve the prediction accuracy and convergence speed of BPNN to the evaluation results of instructional quality.

The article "Construction of Teaching Mode of Film and TV Art in Institution of Higher Learning Using Virtual Simulation Technology" was retracted in 2023. Reasons: suspected computer-generated content; unreliable results or conclusions; concerns about the data; concerns about the results or conclusions.

According to the needs, this paper has set up five chapters, and the specific chapters are arranged as follows: the first chapter is the introduction of the article. This part introduces the research background and corresponding challenges of this paper, and states the significance and innovation of this paper. The second chapter is the literature review part of this paper. This chapter mainly introduces the virtual simulation technology and the related content of film and TV art teaching in institution of higher learning, and summarizes the related research at home and abroad. This leads to the research work and methods of this paper. The third chapter is the research and design part of the article. It mainly provides strategies for art teaching in institution of higher learning and puts forward a new teaching mode; and the teaching evaluation model is constructed. And the process of design and implementation is given. The fourth chapter carries out the experiment of this research and analyzes and discusses the research results in detail. The fifth chapter is the conclusion. Firstly, this chapter summarizes the content of this paper, combing the main conclusions and innovations of this paper; then, it explains the deficiency of the research and the future research direction.

## 2. Related Work

Saraswat et al. believe that virtual education can be applied to a variety of professional education. Different educational content can be customized according to different professional needs. The occupational content is completely different, but the production process of the instructional content is basically the same; it includes the creation of the instructional model, the introduction of the instructional model, and additional instructional actions [8]. Xu et al. proposed that relevant personnel should give full play to the aesthetic education function of film and TV art education in institution of higher learning, correctly understand the industrialization of education, regulate its utilitarian and commercialization issues, improve the quality of teachers, and innovate professional curriculum systems, its connotation and level, and promote the better and faster development of film and TV art education in institution of higher learning [9]. Yubao and others believe that the use of virtual simulation experiment teaching can allow students to improve their professional practice ability in an immersive state, thereby promoting the overall quality of film and TV media teaching [10]. For the purpose of cultivating artistic talents, Zhang et al. discussed the introduction of the virtual simulation platform of artistic cultural heritage into the practical teaching of art majors in institution of higher learning, in order to make up for the shortcomings and deficiencies of practical teaching links, and improve the innovative practice ability of art majors [11]. Bourdeau et al. put forward corresponding solutions to the problems existing in film and TV art education, and clarified the future development direction of virtual simulation technology in art teaching, providing a useful theoretical reference for art design teaching [12].

The article "Construction of Teaching Mode of Film and TV Art in Institution of Higher Learning Using Virtual Simulation Technology" was retracted in 2023. Reasons: suspected computer-generated content; unreliable results or conclusions; concerns about the data; concerns about the results or conclusions.

In the process of establishing a teacher's teaching evaluation system, Wang et al. mainly considered different disciplines and majors, set up different evaluation index items, and established different evaluation index systems [13]. Setiawan et al. analyzed the advantages and disadvantages of previous instructional quality evaluation methods and summarized the problems existing in the current instructional quality evaluation system in institution of higher learning. On this basis, the limitations of the existing instructional quality evaluation system in a university are improved to form a more scientific and reasonable instructional quality evaluation system [14]. Liu et al. established a mathematical model of the instructional quality evaluation system using NN (neural network) theory [15]. After the training of the network, the model can evaluate the instructional quality and provide a meaningful reference value for the research of the instructional quality evaluation system. The improved algorithm based on BPNN proposed by Villanueva et al. provides a scientific and reasonable tool for teaching management in institution of higher learning [16]. The application of this algorithm is highly scientific and rigorous. Shen et al. used adaptive mutation GA to optimize the BPNN model to learn prior sample knowledge and establish an evaluation model. This model reduces the subjectivity of BPNN learning samples [17]. Jong et al. used the feed-forward NN method of BPNN to establish an instructional quality evaluation model, and learned and trained the network through the MATLAB toolbox [18]. Verified by the test data, the results are relatively accurate.

The article "Construction of Teaching Mode of Film and TV Art in Institution of Higher Learning Using Virtual Simulation Technology" was retracted in 2023. Reasons: suspected computer-generated content; unreliable results or conclusions; concerns about the data; concerns about the results or conclusions.

Based on the predecessors' research on virtual simulation technology and the teaching of film and TV art in institution of higher learning, and considering the current learning situation of students majoring in film and TV art, this paper puts forward corresponding teaching methods and modes. In addition, this paper constructs an instructional quality evaluation model to evaluate the feasibility of the teaching model. The evaluation model quantifies the subjective factors in the existing evaluation system and uses NN's self-learning, self-adaptation, and nonlinear approximation capabilities to calculate the quantitative evaluation. Finally, this paper analyzes the algorithms used in the model theoretically and compares the training results. The experimental results show that the algorithm in this paper has certain superior performance, and the teaching mode in this paper is feasible and effective.

## 3. Methodology

### 3.1. Present Situation of Film and TV Art Teaching in Institution of Higher Learning

Film and TV art, from its own nature, has artistic aesthetic function. The integration of art appreciation teaching and classroom should emphasize certain ways and means. On the one hand, it is necessary to match the teaching materials with the film and TV works, so that students can learn by referring to the film and TV works and the contents of the teaching materials, deepen their understanding and mastery of the film and TV art methods, and accumulate experience and materials. On the other hand, teachers should provide students with classic film and TV works, and encourage students to improve their appreciation ability and cognitive level through independent appreciation, group cooperation appreciation, and joint appreciation between teachers and students. However, with the deepening of marketization and the increasing frequency of international exchanges, its market function also occupies a dominant position. These two functions are leading the development of film and TV art, especially in the teaching of film and TV art. Schools, teachers, and students will face a dilemma in these two aspects. Film and TV art is a comprehensive subject that includes many disciplines, and it is also widely used in many fields because of its diversity. However, at present, institution of higher learning usually put too much emphasis on the teaching of several hot majors when constructing such majors. On the one hand, this unbalanced development situation makes students' future employment choices have certain limitations; on the other hand, it is not conducive to improving the overall quality of film and TV art education in institution of higher learning. Teachers are the leader of classroom teaching, leading the style and direction of classroom. College film and TV art teachers should not only have rich theoretical knowledge and profound artistic accomplishment, but also have exquisite teaching methods and classroom control ability. The traditional teaching mode is carried out in the form of teachers' speaking and students' listening, with a single form and boring content. Many contents cannot be effectively presented, which reduces the teaching effect.

The article "Construction of Teaching Mode of Film and TV Art in Institution of Higher Learning Using Virtual Simulation Technology" was retracted in 2023. Reasons: suspected computer-generated content; unreliable results or conclusions; concerns about the data; concerns about the results or conclusions.

At present, many teachers' teaching content is ok on the whole, but it is far from enough in terms of knowledge transfer and depth and breadth. More teachers' teaching methods in class are just classroom lectures, which do not give prominence to students' dominant position. If teachers only instill the boring theory of film and TV art, it will seriously affect students' learning enthusiasm and initiative, and lead to a significant decline in students' independent inquiry ability. At present, with the exception of a few specialized colleges established on the scale of schools with relatively perfect teaching systems, most institution of higher learning is still in the stage of research and exploration on the scientific teaching mode of film and TV art majors, and students are usually evaluated by inherent methods, or the teaching elements cannot really complement each other. Moreover, the traditional teaching of film and TV art in institution of higher learning has the problem of lack of teaching content, which leads to a very single learning resource for students and affects students' comprehensive understanding and grasp of film and TV art. At present, the professional curriculum of film and TV art is still at the stage of exploration and formation. At the same time, the major of film and TV media art has strong applicability, high proportion of practice, great dependence on experimental equipment space, and relatively weak interaction in teaching. This has led to the rapid development of the film and TV art major, and its demand is constantly increasing. Therefore, it is necessary to build an innovative education model.

### 3.2. The Teaching Mode of Film and TV Art in Institution of Higher Learning Based on Virtual Simulation Technology

Virtual simulation technology [19, 20] has the following characteristics:

① Perception of virtual simulation technology
② Specificity of virtual simulation technology
③ Interaction of virtual simulation technology.

The article "Construction of Teaching Mode of Film and TV Art in Institution of Higher Learning Using Virtual Simulation Technology" was retracted in 2023. Reasons: suspected computer-generated content; unreliable results or conclusions; concerns about the data; concerns about the results or conclusions.

Virtual technology can provide an interactive environment for learners, and through the human-computer interface, learners can interact with this environment from the level of personal spiritual feeling. Simulation, on the other hand, extracts an abstract model from the original real system, which can not only truthfully reflect the human-computer interaction relationship existing in the original system, but also truthfully reflect the static structure and dynamic structure of the system. In the past, the fixed and single teaching mode of film and TV art was obviously insufficient in innovation quality. This reflects the limitations of the single teaching mode. Virtual simulation refers to the high degree of human-computer interaction formed by modern artificial intelligence [21, 22], modern network technology, and modern sensing technology. Virtual experiment teaching can make up for the lack of experimental operation in traditional teaching and make students get a chance of experimental operation and training with high degree of reduction and maneuverability, breaking through the limitations of the objective conditions of online and offline teaching. At the same time, it is necessary to flexibly use a variety of different teaching methods, especially to improve the material carrier of film and TV art teaching, and to build multimedia classrooms, simulation studios, audition rooms, etc., so as to provide necessary support for the construction and application of teaching models. The development process of virtual teaching platform and instructional resources is shown in Figure 1.

In the field of art design, it has cross characteristics. The use of virtual simulation technology in art design education can effectively help build a virtual education platform. The virtual platform includes students' training, usual tests, conceptual design of teaching materials, theoretical guidance, user design, and other structures. The effective methods that can be selected in film and TV art education include collective teaching, on-site observation, group cooperation, role simulation, and so on. Different methods have different application scopes, and students' attitudes toward different teaching methods are also very different. In the process of art education, the introduction of virtual simulation technology realizes the perfect combination of virtual technology and art teaching, and makes rational use of various interactive means. In virtual teaching, teachers use advanced technology to help students cultivate their innovative ability. By simulating special effects scenes, scheduling actors, and virtual cameras, the traditional audio-visual language analysis practice that can be completed through two-dimensional media and imagination becomes more stereoscopic and intuitive; it can make students learn the audio-visual language application of different plots more vividly and concretely from different angles.

The article "Construction of Teaching Mode of Film and TV Art in Institution of Higher Learning Using Virtual Simulation Technology" was retracted in 2023. Reasons: suspected computer-generated content; unreliable results or conclusions; concerns about the data; concerns about the results or conclusions.

Various virtual simulation education platforms can be effectively established through the use of virtual simulation technology. Students can use this platform to create works of art based on their own ideas and intentions. Students can use a virtual simulation experiment to preview and virtually restore classic film clips, compare and analyze them over and over, and conduct unlimited studies and research. This will not only improve the quality of instruction in the film and television media major, but it will also encourage students to gain experience and early accomplishments in preparation for actual shooting, as well as deepen their research and thinking abilities. The appropriate application of virtual simulation technology in the art education process benefits all types of virtual laboratories, including mold design and manufacturing, and art decoration laboratories. Immersion, fidelity, interactivity, and imagination are all advantages of virtual experiment teaching, which is experimental and exploratory. Teaching methods and means are elements that require special attention when constructing the teaching mode of film and television art in institutions of higher learning, and they will also have a significant impact on how the teaching mode is implemented in the future. This necessitates college professors paying close attention to summarizing scientific and effective teaching methods in both classroom practice and educational research. At the same time, teachers play a critical role in constructing the teaching mode of film and television art in higher education institutions. We can only ensure the smooth development of teaching work if we have an excellent team of teachers. While preaching, teaching, and dispelling doubts, excellent teachers can provide internship positions and practical opportunities for students.

### 3.3. Construction of Evaluation Model of Film and TV Art Teaching Mode in Institution of Higher Learning

BPNN is a nonlinear dynamic system composed of a large number of processing units. It has excellent learning, memorizing, and calculating abilities. To some extent, this system can imitate the working principle of the brain for information processing. BPNN identifies the evaluation system, and its basic idea is the least square method. Gradient search technique is adopted to minimize the root mean square error between the actual output value and the expected output value of the network. The learning process of network is the process of correcting the weighting coefficient while the error propagates backward, so it can be used to identify the instructional quality evaluation system. The BPNN structure is shown in Figure 2.

The article "Construction of Teaching Mode of Film and TV Art in Institution of Higher Learning Using Virtual Simulation Technology" was retracted in 2023. Reasons: suspected computer-generated content; unreliable results or conclusions; concerns about the data; concerns about the results or conclusions.

The primary task of instructional quality evaluation is to establish an index system of instructional quality evaluation, which should be complete; that is, each index complements each other and constitutes a complete whole. From the perspective of teaching philosophy, teaching should pay attention to the all-round development of students' knowledge, ability, and quality; from the point of view of teaching content, the teaching content should keep close contact with the development of discipline, economy, and society. From the perspective of teaching methods, teaching and training methods should have strong scientific research characteristics, and attention should be paid to cultivating students' spirit of criticism and exploration. Therefore, based on the summary of the research theory and practice of instructional quality evaluation in institution of higher learning, this paper establishes the evaluation index system of instructional quality in institution of higher learning as shown in Table 1.

The index system of this paper has the following characteristics:

① The content is intuitive and concise, easy to understand, and easy for evaluators to make judgments.
② Comprehensive.
③ The evaluation results are reliable and convincing.

Combined with network performance, three-layer BPNN is selected. When determining the number of hidden nodes, too few or too many hidden nodes will affect the network's ability to obtain information, generalization ability, and training time. The formula is as follows:

(1) $$\begin{array}{c} m=\sqrt{n+1}+\alpha ,\\ m=\log\;2^{n},\\ m=\sqrt{n1}. \end{array}$$

Among them, *m* is the number of hidden layer nodes; *n* is the number of input layer nodes; 1 is the number of output layer nodes; and *α* is a constant between 1 and 10. In this paper, the number of hidden layer nodes is determined to be 6 based on the trial and error method.

The 16 evaluation indicators are used as input vectors, which are represented by *X*=(*X*_1_, *X*_2_, *X*_3_,…, *X*_16_, ); the hidden layer nodes are represented by *Y*=(*Y*_1_, *Y*_2_, *Y*_3_, *Y*_4_, *Y*_5_, *Y*_6_) as vectors. *Z*=(*z*) represents the output vector, according to the properties of the excitation function; then,

(2) $$\begin{array}{c} Z\in \left(0,1\right). \end{array}$$

Convert the actual output data of the training set to the numerical value of [0,1], as the expected output, which is represented by the vector *D*=(*d*_1_). The weight from the input layer node to the hidden layer node is

(3) $$\begin{array}{c} W=\left(w_{11},w_{12},w_{13},\ldots ,w_{256}\right). \end{array}$$

The weights from the hidden layer node to the output layer node are

(4) $$\begin{array}{c} T=\left(t_{11},t_{21},t_{31},\ldots ,t_{61}\right). \end{array}$$

The output of the hidden layer node is

(5) $$\begin{array}{c} Y_{j}=f\left(\sum_{i=1}^{16}w_{ij}x_{i}\right),j=1,2,3,\ldots ,6. \end{array}$$

The output of the output layer node is

(6) $$\begin{array}{c} Z=f\left(\sum_{j=1}^{6}T_{j1}y_{j}\right). \end{array}$$

Among them, *f*(*x*) is the excitation function. Set the fitness function as the reciprocal of each individual's learning error. The learning error is shown in formula (7), and the fitness function is shown in formula (8).

(7) $$\begin{array}{c} E=\frac{\sum_{k=1}^{p}\sum_{j=1}^{l}\left(y_{j}^{k}-o_{j}^{k}\right)}{2}, \end{array}$$

(8) $$\begin{array}{c} \text{Fitness}=\frac{1}{E}. \end{array}$$

Among them, *E* is the learning error; *p* is the number of training samples; and *l* is the number of output nodes; it represents the error of the *k* th sample relative to the *j* th output node.

The article "Construction of Teaching Mode of Film and TV Art in Institution of Higher Learning Using Virtual Simulation Technology" was retracted in 2023. Reasons: suspected computer-generated content; unreliable results or conclusions; concerns about the data; concerns about the results or conclusions.

It is assumed that there are *p* pairs of training samples, the network corresponds to different samples with different errors *E*^*p*^, and its root mean square is used as the total error of the network. The formula is as follows:

(9) $$\begin{array}{c} E_{me}=\sqrt{\frac{1}{p}\sum_{p=1}^{p}{\left(E^{p}\right)}^{2}}. \end{array}$$

Calculate the error signal of each layer:

(10) $$\begin{array}{c} \delta^{0}=\left(d_{p}-o\right)o\left(1-o\right),\\ \delta_{j}^{y}=\delta^{0}w_{j}y_{j}\left(1-y_{j}\right). \end{array}$$

The BPNN weight adjustment formula is

(11) $$\begin{array}{c} \left\{\begin{array}{c} \Delta w_{j}=\eta \delta^{0}y_{j}=\eta \left(d_{p}-o\right)o\left(1-o\right)y_{j},\\ \Delta v_{ij}=\eta \delta_{j}^{y}x_{i}=\eta \delta^{0}w_{j}y_{j}\left(1-y_{j}\right)x_{i}. \end{array}\right.. \end{array}$$

Each component in the weight matrix W and *V* is calculated by the above formula.

Because BPNN has hidden layers in the middle and corresponding learning rules to follow, it can be trained to recognize nonlinear patterns. In the design process, this paper takes into account the nonlinear relationship between the evaluation index and the evaluation target, comprehensively analyzes the evaluation system of instructional quality, fully understands the problems to be solved, combines experience with trial, and selects a better design scheme through an improved experiment.

The article "Construction of Teaching Mode of Film and TV Art in Institution of Higher Learning Using Virtual Simulation Technology" was retracted in 2023. Reasons: suspected computer-generated content; unreliable results or conclusions; concerns about the data; concerns about the results or conclusions.

## 4. Result Analysis and Discussion

In this paper, the improved BPNN model is designed by MATLAB toolbox function. The transfer function of BPNN is tangent sigmoid function, and the training function is trainlm. The target error of the network is 0.01, the maximum number of cycles is 1000, and the learning rate is 0.8. Through the training of all samples, and checking the total error of the network, if it meets the accuracy requirements, the training will be finished. The running parameters of GA are weight change range 0.4, crossover probability 0.6, and mutation probability 0.004 to study the data of 100 randomly selected teachers. In order to ensure the high reliability and effectiveness of teaching evaluation indicators, this chapter carries out several tests. The convergence curve results of the algorithm are shown in Figure 3.

Using BPNN to establish the instructional quality evaluation model, as long as the training data are representative and the training is debugged repeatedly, good simulation results can be obtained. Standardize the scoring data [0, 100] to between [0, 1]. In this paper, the maximum-minimum method, a common normalization method, is adopted, which can well preserve the original meaning of data.  Figure 4 shows the recall results of testing different algorithms.

The results show that this method has a high recall rate. From the data obtained through network training, it can be seen that the improved BPNN in this paper is more scientific and accurate than the previous method. From the perspective of structure realization, the method of adding hidden layer nodes is simpler than that of adding more hidden layers, and its training effect is easier to observe and adjust. Therefore, this paper adopts the method of adjusting the number of hidden layer nodes to change the accuracy and efficiency of the network. In addition, in order to test the effectiveness of the college film and TV art teaching mode based on virtual simulation technology proposed in this paper, the algorithm is used to evaluate it. The evaluation results are shown in Figure 5.

From the evaluation data, it can be seen that the teaching model in this paper is feasible and effective. The model proposed in this paper can accurately determine the teaching effect according to each evaluation index. The test results and expert evaluation results are shown in Table 2.

It can be seen from Table 2 that the error range between the test results and the expert evaluation results is small. The comparison of mean square error of different algorithms obtained by experiment is shown in Figure 6.

BPNN has the characteristics of “similar input and similar output.” To a certain extent, the quantity and quality of training samples determine the final evaluation accuracy of this method. In other words, the more the training samples, the higher the quality, and the more accurate the final evaluation result. The evaluation accuracy of this algorithm is compared with that of the other two algorithms, and the results are shown in Figure 7.

The article "Construction of Teaching Mode of Film and TV Art in Institution of Higher Learning Using Virtual Simulation Technology" was retracted in 2023. Reasons: suspected computer-generated content; unreliable results or conclusions; concerns about the data; concerns about the results or conclusions.

Experiments show that the model can overcome various subjective factors and has strong generalization ability. By inputting each evaluation index into the model, the results can accurately evaluate the comprehensive teaching effect of teachers.

This chapter tests the evaluation model of film and TV art teaching mode in institution of higher learning. From the test results, the performance of the model meets the requirements of the analysis stage. Moreover, the algorithm in this paper has faster calculation time and higher stability. The highest evaluation accuracy rate is 94.31%, which is 6.35%∼10.03% higher than other methods. It can effectively evaluate the teaching mode of film and TV art in institution of higher learning. Moreover, the college film and TV art teaching mode constructed in this paper can stimulate students' interest in learning and can effectively provide certain technical and theoretical support for college film and TV art teaching.

## 5. Conclusions

This paper examines the practical significance, development principles, principles, and construction contents of virtual simulation technology for practical teaching of art majors, as well as the status of film and TV art teaching and virtual simulation technology in institutions of higher learning. It also discusses the anticipated effects of using a virtual simulation experimental teaching environment in the practical teaching of art majors, as well as the teaching mode of film and television art in higher education institutions. This paper also develops an instructional quality evaluation model to assess the teaching model's viability. The entropy method, which can be weighted according to the data itself and has the properties of avoiding artificial subjective factors, is used as the guidance mechanism of NN in order to make the learning process of NN more empirical and avoid prior artificial assumptions. Create an entropy method and adaptive GA optimizing BPNN-based instructional quality evaluation model. Experiments show that this algorithm's evaluation accuracy can reach 94.31 percent, which is 6.35 percent higher than other methods by 10.03 percent. It has the ability to assess the film and television art teaching mode in higher education institutions. It has the potential to effectively provide some technical and theoretical support for film and television art teaching in higher education institutions. Virtual simulation technology, on the other hand, necessitates a significant amount of content, which necessitates sufficient manpower, material resources, and time. As a result, this paper will cover a lot more ground. I plan to improve and perfect the evaluation model and teaching mode in the future so that it can better serve teachers and students' work and studies.

The article "Construction of Teaching Mode of Film and TV Art in Institution of Higher Learning Using Virtual Simulation Technology" was retracted in 2023. Reasons: suspected computer-generated content; unreliable results or conclusions; concerns about the data; concerns about the results or conclusions.

## Figures and Tables

**Figure 1:** Virtual simulation teaching platform and instructional resources development process.

**Figure 2:** BPNN structure.

**Figure 3:** Convergence curve of the algorithm.

**Figure 4:** Recall results of different algorithms.

**Figure 5:** Effectiveness evaluation of teaching mode.

**Figure 6:** Comparison of mean square error of different algorithms.

**Figure 7:** Evaluation accuracy results of the algorithm.

**Table 1:** Evaluation index system of instructional quality in institution of higher learning.

Primary index	Secondary index	Index sequence
Teaching objectives	Clear teaching objectives	X1
	Focus and clarity	X2

Content of courses	Combination of theory and practice	X3
	Innovation capacity	X4

Teaching method	Teaching students according to their aptitude	X5
	Be good at enlightening and guiding thinking	X6
	Ability of expression and processing	X7

Teaching attitude	Be patient and active in answering questions	X8
	Serious and infectious teaching	X9
	Rigorous attitude, keep improving	X10

Teaching organization	Situation of preparing lessons	X11
	Coherence of teaching links	X12

Teaching effect	Stimulate students' interest in learning	X13
	Students' self-study ability	X14
	Comprehensive quality of students	X15
	Students' innovative ability	X16

**Table 2:** Comparison between expert data and test values of NN system.

Sample sequence	Evaluation target	Experimental value
1	0.763	0.759
2	0.741	0.738
3	0.729	0.736
4	0.752	0.741
5	0.776	0.769
6	0.764	0.765

## Data Availability

The data used to support the findings of this study are available from the author upon request.
